# Voice Detection and Music Smart Classroom Teaching Application Based on Mobile Edge Computing

**DOI:** 10.1155/2022/4718421

**Published:** 2022-09-21

**Authors:** Jun Huang, Baoli Zhang

**Affiliations:** ^1^Faculty of Science and Engineering, University of Manchester, Manchester, UK; ^2^The Conservatory of Music of Qingdao University, Qingdao, China

## Abstract

Audio monitoring information technology plays an important role in the application of monitoring systems, and it is an indispensable and important link. Whether intelligent audio monitoring management can be successfully realized, the key is to successfully detect abnormal sounds from a variety of external environment background sounds. The core technology of abnormal sound detection is a pattern classification task. The dimension of features is fixed in the traditional abnormal sound detection model. Such an ordinary solution will lead to a long time-consuming detection process and increase the boundary error. Traditional speech detection is not good enough for sound discrimination in a noisy environment, so this paper proposes an abnormal speech detection technology based on moving edge computing. Aiming at the noisy environment of the music classroom, the determination of objective function should be further optimized. Through the related technology, a certain sound can be quickly identified and analyzed in the music classroom to promote the development of the music wisdom classroom, and music wisdom classrooms can be used as a computer-aided system to help music teachers better grasp the learning situation of students, put forward relevant guidance strategies, improve students' learning enthusiasm, and enhance teachers' teaching efficiency so as to promote the progress of music teaching.

## 1. Introduction

Cloud computing can be used as a big data analysis and processing information platform. It has the characteristics of massive storage management capabilities, strong computational thinking, and dynamic resource scheduling. It provides powerful technology for the learning of Chinese scholars who are rapidly developing society under China's economic construction [1]. However, as traditional cloud computing processing methods have gradually shown signs of decline and do not meet the academic needs of scholars, they are being replaced by more advanced edge computing, adding enhanced functions such as computing, storage, and processing on the wireless network side [2]. That is, the IT service environment and cloud computing technology capabilities are carried out at the edge of the mobile communication network, which enables the localization of enterprise business and the successful short-distance deployment of data transmission, providing all-round support for high-bandwidth and low-latency Internet of Things enterprise business [3]. After continuous research by research institutions, it is predicted that by 2025, nearly 50 billion wireless devices will be wirelessly connected to the network. In the future, more than 50% of Internet users' network data in China will need to be analyzed, sorted, dealt with, and stored in the network edge computing system [4]. The business prospects of computing technology in the enterprise market scale facing network edge computing are huge. This article will make full use of the powerful advantages of mobile edge computing to provide professional technical support for abnormal voice detection and intelligent music teaching [5].

There are still violent terrorist attacks that are a fatal threat to the safety of life and property of every Chinese person, as well as the stability and unity of China's various ethnic groups and other countries. Therefore, this type of security issue will inevitably arouse the great attention of the people [6]. Therefore, many research institutions are vigorously developing monitoring technologies that can protect people's safety to monitor the occurrence of terrorist attacks. Intelligent surveillance systems are widely used in our ordinary lives, but in real life, video surveillance systems lack robustness and reliability [7]. Based on the consideration of the problems in video surveillance, this paper proposes the use of audio on the basis of mobile edge computing algorithms. Video network information technology extracts audio and video in the surveillance environment and performs scene analysis. The first step is to use the audio sensor system to intercept the signal transmitted by the abnormal sound, and the second step is to use the intercepted abnormal voice signal analysis technology to generate and perform accurate and comprehensive analysis and detection of abnormal sound events to achieve real-time audio and video monitoring. In addition to using mobile edge computing for abnormal sound monitoring, this article also proposes the application of mobile edge computing to music smart classroom teaching because the proposed smart classroom technology of mobile edge computing helps students learn independently. Music improves students' interest and efficiency in learning music. They can learn independently, learn with unique characteristics, interact with each other and learn anytime, anywhere, and stimulate students' love for music so as to promote learning effectiveness and improve student learning.

## 2. Related Work

In literature, this article gives a detailed description of a new audio event detection method and classification method. This method is an extended framework based on the fully convolutional neural network of the region. The most significant feature of this method is that the logarithmic gray spectrum of the audio signal is the input. The method has two different steps [8]. The first is to detect the existence of abnormal audio events on the system time axis, and the sliding convolution kernel is one detection scheme that filters the candidate areas of audio events through the system area recommendation network technology, also known as boundary detection [9]. In the second stage, make full use of the pooling method that is very sensitive to the quality of time-frequency information to organize and cooperate all the time domain and frequency domain information resources. The detection activities of these candidate areas are carefully managed and classified one by one. Adjust the boundary of the candidate area slightly [10]. Some research constructs a framework that combines the functions of boundary detection and classification. In the short event detection with unsatisfactory audio effects, we make full use of the convolution and cyclic neural network system to construct a single-phase detection model; in this model, create a unit of information technology extraction of audio data signals as analysis; use one-dimensional convolution extracts valuable social features in the two dimensions of the frequency domain and the time domain. At the same time, the value extracted from the two dimensions of the frequency domain and the time domain in the convolutional neural network system can be used [11]. The information system has been analyzed and researched and integrated. Finally, the loss function is used to reduce the loss and false detection problems caused by the difficulty of audio frame recognition. In order to prevent the edge server and cell users from competing for limited resources and in order to solve the problem of user language loading efficiency, this paper proposes to combine the main server to follow the Stackelberg game analysis model, taking the Acer station and the edge computing system server problem as the enterprise leader takes the small cell network base station as the follower and sets the effect reflected by the small cell as the edge service data, which represents the management efficiency of energy usage calculation [12]. It also shows the utilization of edge servers as a design and computational offload overhead. The literature designed a utility function based on profit and expenditure. We also fully proved that the utility function satisfies all the conditions of the convex function and designed a special calculation algorithm for it. The literature explains in detail the problem of low utilization of edge computing resources during the unloading process [13]. Combining game theory and some classic algorithms helps to effectively allocate limited resources during the unloading process, and it further promotes the maximum system throughput during the unloading process [14]. Save energy consumption and provide strong scientific theoretical support for the research of offloading calculation. The literature introduces a new concept, namely mobile edge computing, which brings computing algorithms and saving and saving information resources to the edge of China's mobile communication networks, enabling it to develop capabilities that meet the strict delay requirements of enterprises in the future Run application system software quickly on user management mobile devices [15].

## 3. Research on the Basics of Mobile Edge Computing and Abnormal Voice Detection Algorithms

### 3.1. Basics of Mobile Edge Computing

After research, it is found that there is a new type of communication method in the wireless network communication method which is the mobile ad hoc network; due to the relatively low cost, the scalability is very good, and the wireless solution is that the mobile ad hoc network is widely used in wireless networks which is the main reason for the application. The router is connected to the required gateway port from the mobile ad hoc network system. Although the physical layer is the bottom network layer in the five-layer network system, it can provide the necessary physical layer network link creation, maintenance, uninstallation, and removal for data transmission. The upper level is called the physical link level. The level mainly includes the media access and logical link control levels. The two systems of the media access control level system and the mobile self-configuration network generally use Figure 1 to show that the carrier perceives multiple actions. As an alternative to using other technologies in collision sensing technology and logical link control, this paper proposes a hierarchical structure of mobile AD hoc network simulation.

Research on the edge detection system by the research institute found that there are generally base stations in the traditional network systems that were backward in the past. Relay devices like this usually do not move easily. The network of relay nodes is suddenly continuously connected, and the relay cannot be connected when communicating again. Therefore, the existing network download protocols (such as RIP and OSPF) are the least suitable for mobile ad hoc systems. Therefore, proposing a suitable routing algorithm for the mobile ad hoc network is the best way for us to study and solve the specific background and network output mode of the mobile ad hoc network.

Under the vigorous promotion of the market economy, many types of network classification management models have emerged at the same time. However, because of the different characteristics of the routing discovery mechanism, there are currently three classification methods: the first type is to arrange routing protocols according to the needs of customers for the network, the second type is a table-driven routing protocol, and the third type is a hybrid routing protocol. After the large-scale deployment of mobile self-organizing network nodes is completed, the OPNET simulation system can output the simulation results in the form of branch graphs.

In Figure 2, the horizontal axis represents the broadcast time, and the vertical axis represents the broadcast information. The first transmission point of the broadcast information is the source node. After the broadcast information is transmitted to the neighbor node, it is transmitted to the neighbor node again. The amount of broadcast information is in an unstable state from 0 to 3 seconds, showing an increasing trend, and it gradually becomes stable at 4 s. The status is approaching, and the distribution of broadcast information is about 1000 randomly distributed virtual nodes. In order to ensure the real-time stability and better connectivity of the network users, the success rate is as high as 90%.

The mobile ad hoc simulation network provides a network foundation for the business needs of information context awareness. In the mobile Internet environment, the actual network topology usually exists in a dynamic and unstable state. In this article, the terminal network signal is set to move at a relatively uniform speed. The size of the data information changes mainly because the important business data type settings cannot be guaranteed to be completely consistent. Here, we have selected two very representative application scenarios through careful research. One is to enhance the realistic scene, and the other is the scene of sports health detection. Types of situational awareness applications are shown in Table 1.

The realistic augmented reality scenes and sports health perception scenes shown in Table 1 can be applied to situational awareness network systems. Based on a large amount of data collected regularly by edge nodes and displayed as image information, the requirements for time delay are relatively high, and the data processing cycle is comparative. From the perspective of global situational awareness, it conducts research and discovery of business data requirements and network identification and at the same time performs reasonable processing of the corresponding network services generated. WiFi, Zigbee, Bluetooth, etc., as widely used mobile ad hoc networks, require reliable communication technology, which is a short-distance high-speed network type. WiFi is currently the most popular wireless communication technology. Although the cost and power consumption are high, in order to ensure effective services, this section introduces the connection of three mobile devices to ad-hoc networks. Choose WiFi as the specific network communication according to the size and bandwidth standard.

Almost all wireless networks have the function of inputting and outputting network data. During communication, there is a purpose to select the transmission speed according to the situation of the network link. Ordinary network servers will take up a lot of data uploading. When distinguishing cloud computing and edge computing, as shown in Table 2, the WAN communication distance of the edge server is closer than that of the cloud server, and because the communication bandwidth is very large, it is best to choose the edge server in the case of small data transmission. It is more reassuring that it is more appropriate to choose a cloud computing server when encountering big data transmission.

### 3.2. Research on the Abnormal Speech Detection Algorithm

Researchers have worked hard and discovered that the main algorithm principle of the abnormal sound event detection network program is a pattern recognition problem. The pattern recognition problem is divided into two main steps. The step is to accurately and quickly identify abnormal sound features with clear discrimination capabilities. The second step is to establish and train a suitable classifier on the basis of accurate extraction. After that, statistical machine learning methods are used to establish simulators and later model training tasks for the effective features extracted by abnormal sounds. The purpose is to deepen the basic skills of learning theoretical knowledge from the known data so that these data knowledge can be used for unknown data. Lay a solid foundation for accurate and efficient forecasting. Therefore, it is necessary to extract the effective characteristics of the ideal sound activity based on the excellent performance of the ideal sound perception effect. The successful construction and training of classification models is our ultimate goal. In recent years, Chinese neural networks have combined feature extraction and pattern classification with deep neural networks. At the same time, a lot of efforts have been made for joint training. However, there are still some problems with the rich variability of audio signal data and insufficient signal samples.  Figure 3 shows the basic theoretical framework of abnormal sound event detection.

Because the network audio output signal is a nonstatic time-varying signal during the detection process, the network audio signal has extremely short-term stability. Generally, it is stable in a short period of time, but it is abnormal for a long time. Therefore, in audio signal processing, the core stage is to use the window function to meet the requirements of short-term signal data according to the frame and then perform related processing on each frame of the signal data. The average energy of the audio signal *x* (*n*) is defined as

(1) $$\begin{array}{c} \begin{array}{c} E_{n}=\overset{N-1}{\underset{n=0}{\sum }}x{\left(n\right)}^{2}w\left(n\right)\text{,}\\ M_{n}=\overset{N-1}{\underset{n=0}{\sum }}\left|x\left(n\right)\right|w\left(n\right) \end{array}\text{.} \end{array}$$

At first, the discrete Fourier transform after winding and framing each sound segment. For each segment of the audio signal *x* (*n*), the discrete Fourier transform has its corresponding transform, as shown in the formula:

(2) $$\begin{array}{c} \begin{array}{c} X_{t}\left(k\right)=\overset{N-1}{\underset{n=0}{\sum }}x\left(n\right)w\left(n\right)e^{-2\pi ikn/N},k=0,1,\ldots ,N-1\text{,}\\ S_{Linear}\left(k,t\right)=\left|X_{t}\left(k\right)\right|\text{,}\\ S_{\log}\left(k,t\right)=\mathrm{Log}\left(\left|X_{t}\left(k\right)\right|\right)\text{,}\\ G\left(k,t\right)=\frac{S\left(k,t\right)-\min\;\left(S\right)}{\max\left(S\right)-\min\;\left(S\right)}\text{.} \end{array} \end{array}$$

The output *Y* represents the category of the sample, then the perceptron can be expressed as

(3) $$\begin{array}{c} y=sign\left(w∙x+b\right)\text{,} \end{array}$$

sign is a sign function

(4) $$\begin{array}{c} sign\left(x\right)=\left\{\begin{array}{cc} +1\text{,} & x\geq 0\text{,}\\ -1\text{,} & x<0 \end{array}\right.\text{.} \end{array}$$

The logistic regression model is actually a type of logarithmic linear model. There is a big difference between logistic regression and perceptron. Logistic regression is a conditional probability distribution that satisfies the following equation:

(5) $$\begin{array}{c} \begin{array}{c} P\left(Y=1|x\right)=g\left(w∙x+b\right)\text{,}\\ P\left(Y=0|x\right)=1-g\left(w∙x+b\right) \end{array}\text{.} \end{array}$$

Sigmoid function.

(6) $$\begin{array}{c} g\left(z\right)=\frac{1}{1+e^{-z}}\text{.} \end{array}$$

When *k* = 1, softmax regression is logistic regression, and the loss function of softmax regression is the cross-entropy loss function, which is expressed as follows:

(7) $$\begin{array}{c} h^{1}=f\left(w^{h^{1}i}∙x+b^{h^{1}i}\right)\text{.} \end{array}$$

Generally, when training a neural network system model, a loss function is often used to evaluate the results of the model's prediction of the sample. Common loss functions are

0-1 loss function.

(8) $$\begin{array}{c} L\left(y,f\left(x\right)\right)=\left\{\begin{array}{cc} 0\text{,} & y\neq f\left(x\right)\text{,}\\ 1\text{,} & y=f\left(x\right) \end{array}\right.\text{.} \end{array}$$

Mean square error loss function:

(9) $$\begin{array}{c} L\left(y,f\left(x\right)\right)=\frac{1}{2}{\left(y-f\left(x\right)\right)}^{2}\text{.} \end{array}$$

Log loss function:

(10) $$\begin{array}{c} L\left(y,P\left(y|x\right)\right)=-\log\;P\left(y|x\right)\text{.} \end{array}$$

The discrete form of convolution can be defined as

(11) $$\begin{array}{c} h\left(n\right)=f\left(n\right)*g\left(n\right)=\overset{+\infty }{\underset{m=-\infty }{\sum }}f\left(m\right)g\left(n-m\right)\text{.} \end{array}$$

The forward propagation from the input layer to the hidden layer in the recurrent neural network is shown in the following formula:

(12) $$\begin{array}{c} s\left(t\right)=f\left(V∙x\left(t\right)+U∙s\left(t-1\right)+b^{si}\right)\text{.} \end{array}$$

Table 3 refers to the results of each category of the system in the statistical analysis test data set. In the entire test set, the *f*-score is 70.0%; the ER value is 0.60; it means no. For the baby cry category, the *p*value is much lower than the *R* value, and the FP statistic is much larger than the FN statistic, indicating that many environmental background noises are identified as baby cry, which can be seen by the high IR value. Yes, the ER value is mainly affected by the IR value. In the category of glass breaking, the Dr. value mainly affects the ER value, but it is better than the other two abnormal noise events. The perception of glass breaking is optimistic, and only part of it is perceived as background sound. It can be seen that the Dr. value and IR value are relatively high in the gunshot category, indicating that the baseline method has a weak ability to distinguish between gunshots and environmental background sounds, which is the worst of all categories.

Table 4 shows statistics of the results of the extended r-fcn method (e-rfcn) in each category of the test data set. In the entire test set, the *f*-score is 91.4%, which is 21% higher than the baseline system; the ER value is 0.16, which is obviously higher than the baseline system, and the lower the IR value, the higher the accuracy of environmental background sound recognition; the SR value is almost 0, indicating that there is almost no misrecognition among various abnormal sound events.

Figure 4 shows a sample of baby cry. Since the ultimate goal of the model is to classify the audio signal in each frame, the audio signal in each frame has 4 scores. Each score indicates that the audio signal belongs to the background and the gun. Each score represents the probability that the audio signal belongs to gunshot, glass break, and baby crying. The category in each frame of the audio signal is usually represented by the blue column of the probability map. The actual label of the audio signal is usually indicated by the red line. The boundary created by the probability is automatically predicted to produce green. Different audio signals display different histogram probability graphs, and the size of the probability boundary is also different.

As shown in the left image in Figure 4, most of the frame of the audio signal segment is relatively easy to identify. After converting from 0 to 2, the loss weight value of the audio frame that is easy to identify is reduced. Therefore, in the right image of Figure 4, the predicted probability of the relatively easy-to-recognize part of the background sound will be reduced, but it will not affect the final perception result.

## 4. The Practice of Wisdom Classrooms in Music Teaching

### 4.1. Exploration of the Structure of Music Teaching under the Concept of Smart Classrooms

The music subject itself is learned by learners as an auditory art. The biggest focus of people's attention is that learners learn the main body of music so as to express and regulate people's various emotions. The well-known music itself includes pitch, melody, beat, rhythm, timbre, and so on. Listening is the most effective and basic learning method for music teaching. Newborn children are relatively young, their five senses are in the development stage, and they are more sensitive to voice response and listening. As long as they have a voice, they can attract their attention. Often, the effect of music education and teaching from a baby is significant.

The subject of music is a subject with a strong sense of rhythm, with very significant characteristics. The rhythm itself is abstract, and we generally cannot express it clearly in a concrete form. In the practice of music teaching, we are trying to show the rhythm and rhythm of music songs in a vivid, intuitive, and visible form in front of people. How should we choose the teaching method? The method of classroom practice teaching through rhythmic accompaniment is worth recommending and implementing. Rhythm accompaniment is a kind of music teaching method in which educators use body movements to express the rhythm of music when teaching music. Let every part of the body move with the music street beat, and the students' perceptual thinking and sports thinking will be inspired accordingly, and teaching activities and learning activities will become relatively easy.

As the famous educator Usinsky said, “Comparison is the basis of all understanding and thinking. Only through comparison can we understand everything in the world.” No matter what kind of song, they have their own unique melody, rhythm, and tone. In the ordinary teaching process, if the teacher just blindly teaches in the way of telling, it will not be able to arouse the imagination and interest of the students, the students will feel bored, and the characteristics of the rhythm of the song will not be able to exert its maximum effect. Compared with appreciating music, it is to put two songs with obvious differences together. When analyzing the beat, image, and melody in a comprehensive tone, you should be fully familiar with the characteristics and attributes of the two songs. When comparing the rhythm, pitch, and melody of two songs, students' perceptual thinking is more active, and they can quickly grasp the core of the song and accurately grasp the most important lifeline of the music.

Singing songs is the only important thing in the form of music teaching. Due to the individual differences in the student population, music singing teaching should be taught in accordance with their aptitude and should be different from person to person, innovating a variety of alternative teaching methods. The different performance forms of the chorus, duet, and vocal performance bring different feelings and experiences to students, and it is worthy of a bold attempt by the majority of music educators. The two learning performance methods of chorus and duet singing are more traditional than other forms of singing. Only a single singing method brings students a very low sense of freshness and excitement, which can no longer meet the learning needs of current students. The performance of the song has more content, including the display of the song content and the song design action. A stronger sense of the picture will have a deeper impact on students' thinking. Performances and songs must not only be faithful to the song itself but also be based on it. New content must be integrated. Therefore, the teacher gives the students enough time and space to allow the change of thinking to happen quickly. Singing, as a kind of performance, deepens the expression of feelings while singing, and the artistic expression of students is gradually formed in performance training.

### 4.2. Exploration of Effective Teaching Strategies in Music Smart Classrooms

Teaching reform and optimization under the concept of smart classrooms are gradually applied to the practice of music teaching. Teachers act as guides to stimulate their motivation and initiative in learning so that students can learn better and learn faster in a relaxed and active atmosphere. Deep learning can effectively promote the improvement of students' comprehensive quality of music. In classroom teaching, teachers should establish a teaching model that always takes students as the main body, allowing students to be the masters of the classroom, participating in classroom teaching, allowing students to achieve greater development in active learning, and achieving the establishment of high-quality classrooms.

In a harmonious learning atmosphere, students can play active thinking, explore knowledge in depth, and enable them to creatively understand and master knowledge. In music teaching, teachers should establish an equal relationship with students and make full use of teaching wisdom to organize teaching activities. In classroom teaching where teachers and students participate together, students are more interested in learning. They can participate in performances boldly and actively and learn to sing in combination with performances. In the active classroom atmosphere, the students deepened their understanding of songs and stimulated their feelings of caring for animals.

Learning in the imagination can enable our students to achieve economic development in innovative ways of thinking, explore the professional knowledge they have learned in a diversified and multi-angle manner, and deepen their understanding of music and cultural knowledge. In the process of imagining, students imagined a variety of scenes and stories, developed their innovative design thinking so that they have a deeper understanding of the content of song teaching, experience the beauty of nature, and fully experience the art and culture of learning music charm. Through imagination, teachers can ask students to draw what they imagine. In the happy painting process, students can use color brushes to draw their imagination. In the unique Chinese-characteristic imagination and painting activities, students can give full play to our own creativity and draw through a variety of content so that classroom education and teaching can be carried out in an active atmosphere and show the light of wisdom in more ways.

In music teaching, teachers should make full use of the emotions of students to show the artistic charm of music in the classroom, such as singing the songs they want to teach and playing the musical instruments they are good at. When teachers demonstrate their musical talents, students can use the teacher as a learning example, generate learning motivation to learn music, and actively participate in music learning. After students have exerted their own learning initiative, teachers should pay attention to their learning development and provide them with timely help and guidance so that they can accelerate their understanding of music culture knowledge and improve the comprehensive management ability of Chinese music education. In the learning stage, teachers should encourage and praise students more, stimulate their motivation to learn so that they can rely on their own abilities and master music skills to learn, and effectively master the content of learning. When students have some negative emotions, teachers should promptly educate and guide them so that their negative emotions can be expressed, establish students' positive attitude towards learning and life, actively develop thinking in learning, and effectively master the content of music teaching materials. Through the effective guidance of teachers, students can be integrated into the teaching system, play their own strengths, exercise their abilities, and promote the progress of the music teaching level. Therefore, teachers play a guiding role in this system and guide students to study independently, actively participate in learning activities, and deepen their understanding and experience of music through imagination and exploration. In teaching practice activities, teachers should create a good relationship between teachers and students, provide students with a harmonious learning environment for development so that they can conduct in-depth exploration under the guidance of teachers, master effective learning and research methods, and think through. With a solid knowledge of music culture, you can improve your ability to explore music, complete your own learning-related content efficiently, and create a high-quality music classroom.

## 5. Conclusion

Aiming at the current problem of excessive information, the application of mobile edge computing can alleviate various problems caused by excessive information to traditional cloud computing to a certain extent, reduce the lag of cloud computing in processing information, and reduce the energy consumption in the process of processing information to relieve the pressure of the network center. The research shows that the moving edge computing algorithm proposed in this paper can alleviate the related pressure of data processing and improve the accuracy of data processing. This article applies mobile edge computing to abnormal speech detection and music wisdom classroom teaching. With the development of security monitoring technology, abnormal noise detection has attracted more and more attention. At present, most research methods in China are based on traditional Chinese speech recognition methods. Therefore, in this article, we can use the edge of China's mobile network to perform our research on abnormal sound recognition. In order to better promote the development of abnormal speech detection in music classrooms and promote the application of the system, this paper also analyzes the commercialization of abnormal speech detection at home and abroad, analyzes the difficulties in the research and teaching of abnormal sound detection, and explains the main learning content of this article. A smart classroom is used to enrich the content of the classroom. Teachers are good at using various forms to increase the attractiveness of the classroom to students so that students can learn and grow healthily under the guidance of the teacher. Teachers and students sing with music tables to express true emotions and effective interaction, which creates a good learning atmosphere for the establishment of a harmonious social relationship between teachers and students.

## Figures and Tables

**Figure 1:** CSMA/CA (carrier sense multiple access technology with collision detection).

**Figure 2:** Relationship between OLSR broadcast information and time.

**Figure 3:** The basic framework of abnormal sound event detection.

**Figure 4:** Test results of a music. (a) *γ* = 0. (b) *γ* = 2.

**Table 1:** Types of situational awareness applications.

Parameter application	Augmented reality	Mobile health awareness
Edge node mobility mode	Larger range of movement	Smaller range movement
Type of data	Image information	Numerical information
Delay demand	Relatively high	Relatively low
Data processing cycle	Relatively short	Relatively short
Quantity	Many	Less

**Table 2:** Cloud and edge comparison table.

Type	Cloud	Edge
Computing power	Strong	Stronger
Communication type	Wan	Wireless local area network
Communication distance	Far	Near
Communication cost	High	Low
Transmission delay	High	Low

**Table 3:** Results of the baseline system in each category.

Class	F (%)	P (%)	R (%)	ER	DR	IR	SR
Baby cry	69.5	60.1	82.4	0.72	0.18	0.55	0.00
Glass break	88.1	93.7	83.2	0.22	0.17	0.06	0.00
Gunshot	51.2	60.3	44.4	0.85	0.56	0.29	0.00
All	70.0	70.1	70.0	0.60	0.30	0.30	0.00

**Table 4:** Results of the E-RFCN method in each category.

Class	F (%)	P (%)	R (%)	ER	DR	IR	SR
Baby cry	97.2	97.1	97.2	0.06	0.03	0.03	0.00
Glass break	94.6	98.7	80.4	0.10	0.09	0.00	0.01
Gunshot	81.4	90.3	75.6	0.32	0.28	0.04	0.00
All	91.4	94.1	82.17	0.16	0.13	0.02	0.01

## Data Availability

The data used to support the ﬁndings of this study are available from the corresponding author upon request.
